# Sustainable fashion: Design of the experiment assisted machine learning for the environmental-friendly resin finishing of cotton fabric

**DOI:** 10.1016/j.heliyon.2023.e12883

**Published:** 2023-01-10

**Authors:** Md Nahid Pervez, Wan Sieng Yeo, Faizan Shafiq, Muhammad Munib Jilani, Zahid Sarwar, Mumtahina Riza, Lina Lin, Xiaorong Xiong, Vincenzo Naddeo, Yingjie Cai

**Affiliations:** a Hubei Provincial Engineering Laboratory for Clean Production and High Value Utilization of Bio-based Textile Materials, Wuhan Textile University, Wuhan 430200, China; b School of Computing, Huanggang Normal University, Huanggang 438000, China; c Sanitary Environmental Engineering Division (SEED), Department of Civil Engineering, University of Salerno, Fisciano 84084, Italy; d Department of Chemical and Energy Engineering, Faculty of Engineering and Science, Curtin University Malaysia, CDT 250, 98009 Miri, Sarawak, Malaysia; e Department of Textile Processing, National Textile University, Faisalabad, Punjab 37610, Pakistan; f School of Engineering and Technology, National Textile University, Faisalabad, Punjab 37610, Pakistan; g Department of Applied Ecology, North Carolina State University, Campus Box 7617 Raleigh, NC 27695-7617, USA

**Keywords:** Resin finishing, Sustainability, Free formaldehyde, Taguchi, Machine learning

## Abstract

Given the carcinogenic properties of formaldehyde-based chemicals, an alternative method for resin-finishing cotton textiles is urgently needed. Therefore, the primary objective of this study is to introduce a sustainable resin-finishing process for cotton fabric via an industrial procedure. For this purpose, Bluesign® approved a formaldehyde-free Knittex RCT® resin was used, and the process parameters were designed and optimized according to the Taguchi L_27_ method. XRD analysis confirmed the crosslinking formation between resin and neighboring molecules of cotton fabric, as no change in the cellulose crystallization phase. Several machine learning models were built in a sequence to predict the crease recovery angle (CRA), tearing strength (TE) and whiteness index (WI). Assessment of modelling was evaluated through the use of various metrics such as root mean square error (RMSE), mean absolute error (MAE), and the coefficient of determination (R^2^). Results were compared to those from other regression models, such as principal component regression (PCR), partial least squares regression (PLSR), and fuzzy modelling. Based on the results of our research, the LSSVR model predicted the CRA, TE, and WI with substantially more accuracy than other models, as shown by the fact that its RMSE and MAE values were significantly lower. In addition, it offered the greatest possible R^2^ values, reaching up to 0.9627.

## Highlights

• A novel combined DoE and machine learning approach was applied.
• Bluesign® approved a formaldehyde-free sustainable Knittex RCT® resin was used.
• Process parameters were designed and optimized by the Taguchi design (L_27_).
• The predictivity assessment of the responses was computed with machine learning models.
• The least-square support vector regression model was the most accurate (R^2^ = 0.9627).

## 1 Introduction

Cotton's adequate air permeability, mechanical characteristics, softness, and comfort ensure that it continues to be the most widely used natural cellulose fabric globally, despite the proliferation of synthetic textile fibers. Cotton, on the other hand, has a tendency to wrinkle, which, in comparison to the properties of many polymers, restricts its use in applications involving public protection and draws attention away from its viability as a material for clothing [[1], [2], [3], [4]].

To address this issue, scientists have turned to utilize a commercially available multifunctional crosslinker to settle the hydroxyl groups of the cellulose next to one another [5]; this is often done using N-methylol compounds like dimethyloldihydroxyethylenurea, a well-known resin finish [6]. Peterson [7] performed a notable review in which he discussed the idea of cross-linking agents, the impact of cross-linking on cellulose fibers, and the existence of a crosslinking reaction occurring inside the cellulose's non-crystalline area. However, resin application alters the interconnecting of the cellulose chains, contributing to the loss of the fabric's rip strength; this is an important concern in many areas. Some scholars have proposed introducing polymer-based modifiers during the finishing process of cellulosic textiles to strike a better balance between the needs for strength in the fabric, cheap cost, and crease resistance. Researchers have created a way of utilizing formaldehyde-free crosslinking agents for the cotton fabric to replace the conventional N-methylol reagents, including zero formaldehyde-based reactants, the low-cost production of 1,3-dimethylurea and glyoxal, and inorganic phosphates. Due to rising public awareness of formaldehyde's risks and the subsequent restriction of formaldehyde-based finishes in many countries, a mitigation procedure, including the development of non-formaldehyde-based resin finishing for crease-resistant textiles, has become necessary [8,9].

As a whole, the performance of the resin finishing process is affected by a wide variety of factors, thus its operations need to be simplified and managed to get optimal results. It is common knowledge that traditional optimization procedures are time-consuming and costly since they require holding all other variables constant while tweaking a single variable [10]. The Taguchi method is one of a kind since it employs analysis of variance (ANOVA) to find statistically significant differences between groups with a minimum of tests. Taguchi trial arrangement helps reduce the expense of trials, improve their quality, and provide solid direction when selecting parameters [[11], [12], [13]]. However, this Taguchi model is unable to provide accurate predictions for process parameters that fall outside the ranges covered by the input data. As for this, machine learning (ML) is being utilized in many disciplines to speed up these procedures and reduce the time and expense of simulation instead of using the conventional statistical Taguchi method [14]. Machine learning models, such as the least square support vector regression model (LSSVR), are capable of learning insights directly from data and understanding how they function with a variety of inputs. In particular, the LSSVR model displays strong predictability to anticipate the desired output variable for nonlinear data. This nonlinear prediction model, called the LSSVR model, is based on the theory of the support vector machine (SVM) [15]. By using a different set of linear equations in a dual space, LSSVR provides a more effective response than the SVM for reducing the computing load associated with reducing the number of possible classes. As a result, throughout the course of many years, scholars from a wide variety of fields paid a growing amount of attention and interest [16].

Consequently, the current study has evaluated the predictive performance of the sustainable resin-finishing process of cotton fabric using the robust LSSVR model integrated with the Taguchi model for the first time. Following that, the precision of the LSSVR is determined by computing the coefficient of determination (R^2^), the root mean square error (RMSE), and the absolute mean error (MAE). In addition, the findings are compared to those produced by using models of the fuzzy model, principal component regression (PCR), and partial least squares regression (PLSR) for a better understanding of their predictive characteristics.

## 2 Experimental

### 2.1 Materials and reagents

Commercial cotton fabric (100% woven) was collected from a local textile factory and chosen for this research with the following parameters in mind: 85 ends per inch (EPI) x 52 picks per inch (PPI), 40 s Ne yarn count, and 102 g/m^2^ fabric weight. Huntsman (USA) supplied both the Knittex RCT® cross-linker and the Knittex® Catalyst Mo, which was employed as the catalyst. Nonionic polysiloxane-based Siligen GL was employed as a softener and collected from BASF in Switzerland. As found, all other chemicals and reagents were of analytical grade during the experimental period.

### 2.2 Design of experiments (DoE) for the resin finishing process

In this investigation, Taguchi's orthogonal array design of experiments (L_27_) is used to design the resin finishing procedure. The data is analyzed using Minitab® 17, a commercial statistical software package [17,18]. The results of the 27 different trials (five variables with three levels) are summarized in Tables S1 and S2 [19,20]. According to the above experimental setup, resin finishing was carried out using a custom-made laboratory methodology using a padder and stenter equipment. Acetic acid was added in a trace amount (three to four drops), sufficient to keep the solution's pH at 5.5 as desired. In accordance with the experimental design, each fabric sample was first padded with a wet pick-up rate of 75%, then dried at a temperature of 120 °C for 3 min, and then cured. After that, the cloth was taken out of the curing chamber, let to cool at ambient temperature, and then ironed.

After that, the fabric samples' crease recovery angle (CRA) was determined using the test method 128–1974 developed by the American Association of Textile Chemists and Colorists. In accordance with the requirements of the ASTM D1424 standard, an intensity tearing tester of the Elmendorf type was used for the tearing strength (TE). The whiteness index (WI) was measured using a HUNTER Lab D25 manufactured in the United States of America following the AATCC Test Method E 313.

### 2.3 Machine learning models development

A total of 27 datasets were adopted from the resin finishing process parameters of cotton fabric, including the concentration of resin (Knittex RCT), polyethylene softener, catalyst (Knittex® Mo), curing temperature, curing time with their responses, namely, crease recovery angle (CRA), tearing strength (TE), and whiteness index (WI). After being imported into MATLAB, the datasets were divided into a training set and a test set, each with an 80:20 split (Table S3). Fig. 1 depicts the overall structure of the regression models (PCR, PLSR, Fuzzy approach, and LSSVR) used to predict CRA, TE, and WI values. The training data are used in the development of models such as PCR, PLSR, the fuzzy approach, and LSSVR, as seen in Fig. 1. In addition, PCR, PLSR, Fuzzy technique, and LSSVR models were used for both the training and testing data, and these same models served as the basis for the assessment of the models' development. All of the different regression models' RMSE, MAE, and R^2^ values were analyzed and compared. Table 1 presents a summary of the parameter settings for the PCR, PLSR, Fuzzy approach, and LSSVR models. The total number of datasets, the number of datasets used for training, the number of datasets used for testing, and the number of latent variables are denoted by the notations NT, N1, and N2 correspondingly. In the meanwhile, the tuning parameters that are employed in the LSSVR model are denoted by the symbols γ, λ, and p.

**Fig. 1:** A framework of PCR, PLSR, Fuzzy method, and LSSVR models.

**Table 1:** Values used for PCR, PLSR, Fuzzy method and LSSVR models.

Parameters	$N_{T}$	$N_{1}$	$N_{2}$	LV	γ	λ	*p*
Values	27	21	6	1	32	0.0625	3.051 × 10^−5^

### 2.4 Prediction behaviour

The root-mean-square error (RMSE) is a scale-dependent defect measure used rather often in evaluating the efficacy of prediction models [21]. This measure was used to test whether or not the data splitting ratio was adequate since it enables comparisons to be made between various configurations for a particular variable. To put it another way, root-mean-square error (RMSE) is a metric that estimates how far a model strays from the true answers, with a smaller number indicating more forecast accuracy. The root square of the sum of the squared discrepancies that exist between the actual output and the predicted output is the RMSE [21]. Alternatively, it may be thought of as an indication of the differences between the predicted and actual values. With that in mind, a smaller RMSE indicates higher accuracy and prediction ability. Equation (1) displays the RMSE formula [22].

(1) $$RMSE=\sqrt{\frac{{\sum_{i}\left(Y_{i}-{\hat{Y}}_{i}\right)}^{2}}{n}}$$

Herein $Y_{i}$ represents the actual output, ${\hat{Y}}_{i}$ is the predicted output, and *n* denotes the total number of samples.

As stated in Equation (2), the MAE is a measurement of the average number of defects in a collection of predictions, and it does not consider the way the errors are pointed. It is the average, calculated across the test sample, of the absolute differences between the anticipated and actual observations, with each individual difference contributing an equal amount of weight to the final result.

(2) $$MAE=\frac{1}{n}\sum_{j=1}^{n}|Y_{i}-{\hat{Y}}_{i}|$$

where ∑ denotes the summation.

R^2^ is a statistic that indicates how effectively a regression model captures a given dataset's share of the total variance [21]. To put it in other words, R^2^ is a measure that tells you how well the actual data fits the anticipated data (also known as “goodness of fit”) in the regression model. Its value may vary anywhere from 0 to 1 [23]. If the number is closer to one, it indicates that most of the output can be expected based on the inputs that have been chosen, which results in a better fit. R^2^ is calculated by contrasting the total number of squared errors with the total number of squared deviations from the mean of the variable in question. R^2^ is a statistical metric that determines how well actual and expected variables match up with one another. The formula in its entirety may be found in Equation (3) [24].

(3) $$R^{2}=1-\frac{{\sum_{i}\left(Y_{i}-{\hat{Y}}_{i}\right)}^{2}}{{\sum_{i}\left(Y_{i}-\bar{Y}\right)}^{2}}$$

Furthermore, the prediction error (PE) is used, and its mathematical representation may be found in Equation (4) [25]. In order to demonstrate the predictive ability of CRAo, TE, and WI in a quantitative manner, the error of approximation, denoted by Ea, is explored, and Ea is calculated using Equation (5) [26].

(4) $$PE=\left|\frac{V_{1}-V_{2}}{V_{1}}\right|\times 100\%$$

(5) $$E_{a}=\left(\frac{N_{1}}{N_{2}}\right){RMSE}_{1}+\left(\frac{N_{2}}{N}\right){RMSE}_{2}+\left|{RMSE}_{1}-{RMSE}_{2}\right|$$

where $V_{1}$ and $V_{2}$ stand for the values that are intended to be achieved and those that are actually accomplished, respectively. *RMSE*_*1*_ and *RMSE*_*2*_ are used to represent the RMSE of training and testing datasets, whilst *MAE*_*1*_ and *MAE*_*2*_ are used to represent the MAE of training and testing datasets.

## 3 Results and discussion

### 3.1 Sustainable resin finishing

Resin application is a common technique used in the textile industry's finishing section to enhance the functional properties of fabrics. Accordingly, the current study evaluated a sustainable resin finishing of cotton fabric using a formaldehyde-free Knittex RCT® resin, approved by Bluesign® (sustainable solution for textiles) [27]. Generally, the cotton fabric crease recovery angle in the resin finishing process is considered one of the most important properties since it determines the fabric recovery folding ability after deformations. Also, the tearing strength of the fabric is a particularly significant quality to consider because of the direct connection that this characteristic has with the fabric's serviceability. If the whiteness value is higher, it means that the cotton fabric has a higher degree of whiteness. Before the cotton cloth is dyed, printed, or subjected to any other wet treatments, a whiter appearance is sought. Whiteness value can also be affected during the resin finishing process, as the curing temperature increases, more crosslinking forms in the catalyst, leading to the fabric's less whitening. As can be seen in Fig. 2a, the crosslinking formation between resin and neighboring molecules of cotton fabric [28]. The molecules of the fibers are less likely to shift position under stress thanks to crosslinking, which also reduces the likelihood of shrinking and wrinkling and improves whiteness. This phenomenon can be correlated with the XRD pattern of untreated and resin-finished fabric (Fig. 2b). Peaks at 2θ of 14.88, 16.48, 22.98, and 34.48° are typical cellulose-I crystallization, as shown in the untreaed fabric [9]. The XRD pattern of resin-finished cotton fabric shows no change in the typical peaks, confirming that the cross-linking utilizing Knittex RCT® does not disrupt the structured crystalline phase of the cellulose [29].

**Fig. 2:** Crosslinking reaction between the cotton fabric and resin product (a) and XRD of untreated and resin-finished fabric (b).

It has been demonstrated that this resin-finishing process's operational parameters might influence end-use performance [30]. As mentioned earlier, Taguchi's design was employed for the resin-finishing process using important parameters, including the concentration of resin, softener, catalyst, curing temperature, and time, which are nonlinear. After that, the parameters of the resin finishing process need to be tuned to determine how effective it is at producing the degree of crease recovery angle, tearing strength, and whiteness required for the cotton fabric.

### 3.2 Feature selection

In this study, the feature selection was performed using principal component analysis (PCA). PCA is a well-known linear feature extractor used for unsupervised feature selection based on eigenvectors analysis to determine critical original features for principal components [31]. In PCA, the variances of the principal components are the eigenvalues of the covariance matrix that illustrates the correlations or relationships between the input variables. Hence, the larger the percentage of the variance, the more important the corresponding variable or it reveals and the more relevant information [32]. The variances for the input variables, including resin (Knittex RCT), polyethylene softener, catalyst (Knittex Mo), curing temperature, and curing time calculated from PCA are 632.0161, 73.2251, 64.7666, 18.2146, and 0.7824, respectively. From these results, it can be concluded that the first four input variables (Resin, polyethylene softener, catalyst, and curing temperature) explain 99.9% of the variation in the data of this study.

Fig. 3 shows a PCA biplot for feature selection of the sustainable resin finishing of cotton fabric. Fig. 3 shows that the four variables, Resin, polyethylene softener, catalyst, and curing temperature, have larger loadings (longer lines). The loadings describe the importance of the independent or input variables and reveal the relationships between variables [33]. Hence, Fig. 3 exhibits similar results as mentioned above in which the first four input variables, resin, polyethylene softener, catalyst, and curing temperature, are important.

**Fig. 3:** A PCA biplot for feature selection of the sustainable resin finishing of cotton fabric.

### 3.3 Modelling assessment

The resin-finishing process parameters may be used in conjunction with predictive modelling tools, such as the LSSVR model, to get estimates of the resin-finished cotton fabric's properties, such as its CRA, TE, and WI. Previously, a few studies have been concerned with modelling the resin-finishing process in the presence of statistical design [34,35]. However, this approach can only provide predictions within the parameters of the provided data. Thus, in this work, various machine learning models, such as LSVVR, Fuzzy method, PLSR, and PCR, were designed to address the shortcomings of this mathematical modelling technique by using the resin finishing process parameters.

For convenience, Tables 2–4 compile the findings of the aforementioned machine-learning models for CRA, TE and WI, respectively. In this study, three popular error metrics, including *RMSE*, *MAE,* and *R*^*2,*^ were used to quantify a model's performance to avoid bias in assessing the model performance [36]. As can be noticed in Tables 2–4, the error metrics for the training data are *RMSE*_*1*_*, MAE*_*1*_*,* ${R_{1}}^{2}$, while *RMSE*_*1*_*, MAE*_*1*_*,* ${R_{2}}^{2}$ are the error metrics denoted for the testing data. According to the data shown in Table 2, the LSSVR model exhibited the highest degree of accuracy for CRA in its predictions, followed by the Fuzzy method, PCR, and PLSR models, particularly those for training data. From Table 2, it can be seen that the *RMSE* and *MAE* values for LSSVR are 25%–304% lower than the Fuzzy method, PCR, and PLSR models, while its R^2^ values are 2%–480% higher.

**Table 2:** Predictive modelling results for CRA from LSSVR, Fuzzy method, PLSR, and PCR.

Models	LSSVR	Fuzzy method	PE (%)	PLSR	PE (%)	PCR	PE (%)
Training data							
*RMSE*_*1*_	1.3043	1.7113	31	3.0720	136	3.0484	134
*MAE*_*1*_	1.0804	1.3524	25	2.3140	114	2.2916	112
${R_{1}}^{2}$	0.9627	0.9425	2	0.7632	21	0.7676	20
Testing data							
*RMSE*_*2*_	1.5247	6.0641	298	2.1035	38	2.0234	33
*MAE*_*2*_	1.1724	4.7333	304	1.5702	34	1.5371	31
${R_{2}}^{2}$	0.9153	−3.4749	480	0.8890	3	0.8960	2
*E*_*a*_	1.5737	7.0314	347	3.8252	143	3.8456	144

**Table 3:** Predictive modelling results for TE from LSSVR, Fuzzy method, PLSR, and PCR.

Models	LSSVR	Fuzzy method	PE (%)	PLSR	PE (%)	PCR	PE (%)
Training data							
*RMSE*_*1*_	9.1384	13.4796	48	17.6421	93	17.9090	96
*MAE*_*1*_	7.0616	10.5524	49	14.5580	106	14.7655	109
${R_{1}}^{2}$	0.9589	0.9238	4	0.8328	13	0.8268	14
Testing data							
*RMSE*_*2*_	11.1836	51.8610	364	18.7417	68	19.0544	70
*MAE*_*2*_	7.2563	46.8000	545	15.9857	120	16.4841	127
${R_{2}}^{2}$	0.9471	−3.7482	496	0.8171	14	0.8069	15
*E*_*a*_	11.6381	60.3901	419	18.9861	63	19.3089	66

**Table 4:** Predictive modeling results for WI from LSSVR, Fuzzy method, PLSR, and PCR.

Models	LSSVR	Fuzzy method	PE (%)	PLSR	PE (%)	PCR	PE (%)
Training data							
*RMSE*_*1*_	0.7786	1.0626	36	1.3688	76	1.3619	75
*MAE*_*1*_	0.6199	0.8524	37	1.0942	77	1.0900	76
${R_{1}}^{2}$	0.7192	0.7808	9	−0.5229	173	−0.4848	167
Testing data							
*RMSE*_*2*_	0.2133	1.5530	628	0.6500	205	0.6351	198
*MAE*_*2*_	0.1646	1.3500	720	0.5278	221	0.5168	214
${R_{2}}^{2}$	0.9585	−1.0549	210	0.6603	31	0.6752	30
*E*_*a*_	1.2183	1.6619	36	1.9279	58	1.9272	58

Moreover, in Table 3, the LSSVR model exhibited the highest degree of accuracy in its TE predictions, followed by the Fuzzy method, PLSR, and PCR models. Again, in Table 3, the LSSVR model shows 48%–545% lower *RMSE* and *MAE* values, as well as 4%–496% higher R^2^ as compared to the Fuzzy method, PCR, and PLSR models. Similarly, for WI displayed in Table 4, the LSSVR model outperformed as compared to the rest of the models, although its R^2^ is slightly lower than the fuzzy method. However, in Table 4, the LSSVR model still provides better overall results since its *RMSE,* and *MAE* values are lowered by 36%–720% compared to the rest of the models. Except for the ${R_{1}}^{2}$ in Table 4, the R^2^ values for the LSSVR model are 30%–210% better than the Fuzzy method, PCR, and PLSR models. From Tables 2–4, the LSSVR model provided the best results due to the additional model in the LSSVR model, namely the leave-one-out cross-validation model that obtained the best tuning parameters for prediction [25]. Furthermore, the radial basis function kernel function used in the LSSVR model, which is a famous kernel function, maps the nonlinear experimental data into a higher dimensional space that can give a better prediction.

On the other hand, from Tables 2–4, notice that the Fuzzy method from the fuzzy logic designer app in MATLAB has better results for the training data. However, for testing data, the fuzzy method gave the worse results since its ${R_{2}}^{2}$ for CRA, TE and WI are negative values, indicating the fuzzy method has a very bad predictive performance. According to Satrio et al. [37], the negative R^2^ values mean the distance from the actual data to the predicted data; from the which is the fuzzy method in this study is very far, and its predicted data are very different and do not match with its actual data. This is because the fuzzy method is developed using a membership function, fuzzy logic operators, and if-then rules based on the training data. These three components involve a selection of fuzzy rules, a database that explains the membership functions used in the fuzzy rules, and a reasoning mechanism that shows the inference way upon the rules to adopt predicted data [38]. As a result, the fuzzy method performs badly when the testing data is different from the training data used for the fuzzy method development.

Despite that, both PCR and PLSR models gave quite similar results in Tables 2–4; even PLSR includes the input and output variables in its model development while the PCR model involves the input variables only [25,39]. Their similar results are due to their assumption that the input variables have the same importance towards the prediction performance [23]. Aside from their similar results, when dealing with the testing data, both PCR and PLSR models performed better than the fuzzy method. This is because PCR and PLSR models are dimension deduction methods that extract independent components from the training data to fit one or more response variables (variables that are required to predict) [40].

### 3.4 Predictivity assessment

Besides evaluating the model's performance using three errors metrics, comparisons of predictive results for CRA, TE, and WI from PCR, PLSR, Fuzzy method, and LSSVR models using the training and testing data were made, as shown in Fig. 4(a)–4(f). In these Fig. 4(a)–4(f), error bars that show the confidence level of actual data or the deviation along a line for the actual curve are included. Fig. 4(a)–4(f) show that the predicted data from the LSSVR model is closer to the actual data than the fuzzy method, PLSR, and PCR models. The closer the predicted data with the actual data, the better the predictive ability of the model [41]. Moreover, in Fig. 4(a)–4(f), the majority of the predicted data from the LSSVR are fallen within the error bars. Besides, it is also noticed that the predicted data from the Fuzzy method are mostly outside the error bars. In conclusion, these figures have double-confirmed that the LSSVR model is the best model for predicting CRA, TE, and WI.

**Fig. 4:** Comparison of predictive results from PCR, PLSR, Fuzzy method, and LSSVR models (a) prediction of CRA using training data, (b) prediction of CRA using testing data, (c) prediction of TE using training data, (d) prediction of TE using testing data, (e) prediction of WI using training data, and (f) prediction of WI using testing data.

### 3.5 Accuracy of the models

The same data sets were used for evaluating the accuracy of the model in terms of coefficients (R^2^). Fig. 5(a)–5(f) reveal the correlation between the actual and predicted values for CRA, TE, and WI from the LSSVR model using the training and testing data. The closer the point to the line, the better the model performance in prediction [42]. From Fig. 5(a)–5(f), it can be noticed that all of the data points are rather close to the line. This suggests that the outputs that were predicted by LSSVR are relatively close to the actual data that were tested for all responses. To some extent, good agreement between the model's predictive values and the actual experimental results is indicative of the model's validity [43]. In conclusion, the LSSVR model is suitable for predicting CRA, TE, and WI, which are essential parameters to optimise the resin finishing performance on cotton fabric.

**Fig. 5:** Correlation between the actual and predicted values from the LSSVR model (a) CRA using training data, (b) CRA using testing data, (c) TE using training data, (d) TE using testing data, (e) WI using training data, (f) WI using testing data.

## 4 Conclusions

To predict the CRA, TE, and WI of resin-finished cotton fabric, the present research established an innovative approach, which was given the combined Taguchi-integrated LSSVR model. This integrated model was constructed using the experimental findings of the resin finishing process with five input variables: concentration of resin (Knittex RCT), polyethylene softener, catalyst (Knittex® Mo), curing temperature, and curing time. In order to get the most CRA, TE, and WI out of the cotton fabric, it is essential to find the resin finishing procedure conditions that work best. As a result, the predictive modelling methods, which may include LSSVR, play a crucial part in the processes used to manufacture resin-finished cotton textiles to achieve the desired level of quality. According to the results, the LSSVR model predicted the CRA, TE, and WI with substantially more accuracy than other models, as shown by the fact that its RMSE and MAE values for LSSVR are 25%–304% lower, 48%–545% lower, as well as 36%–720% lower than the Fuzzy method, PCR, and PLSR models, while its R^2^ values are 2%–480% higher, 4%–496% higher, and 30%–210% better, respectively. Based on these findings, it can be concluded that the LSSVR model has the potential to serve as a predictive model for the resin-finishing process in the textile industry. It is possible that the prediction performance of the LSSVR model might be improved by the use of another algorithm in further research by integrating it. In addition to this, the new characteristics of the process of resin-finishing cotton fabrics, as well as the costs associated with optimizing the process, should get a greater amount of attention. On the other hand, future studies can be done to include more datasets from the experiments to improve the performance of the LSSVR model.

## Author contribution statement

Md. Nahid Pervez: Conceived and designed the experiments; Performed the experiments; Wrote the paper. Wan Sieng Yeo: Analyzed and interpreted the data; Contributed reagents, materials, analysis tools or data; Wrote the paper. Faizan Shafiq: Conceived and designed the experiments; Performed the experiments. Muhammad Munib Jilani, Zahid Sarwar: Performed the experiments. Mumtahina Riza, Xiaorong Xiong: Analyzed and interpreted the data. Lina Lin: Conceived and designed the experiments; Contributed reagents, materials, analysis tools or data. Vincenzo Naddeo: Analyzed and interpreted the data; Contributed reagents, materials, analysis tools or data. Yingjie Cai: Conceived and designed the experiments; Contributed reagents, materials, analysis tools or data; Wrote the paper.

## Funding statement

Yingjie Cai was supported by 10.13039/501100010030China National Textile and Apparel Council (2013‘‘Textile Vision’’ Applied Basic Research, 2013-153).

## Data availability statement

Data will be made available on request.

## Declaration of competing interest

The authors declare that they have no known competing financial interests or personal relationships that could have appeared to influence the work reported in this paper.
